The article "Antiprostate Cancer Activity of Ineupatolide Isolated from Carpesium cernuum L" was published in 2021. Journal: Biomed Res Int.

# Antiprostate Cancer Activity of Ineupatolide Isolated from *Carpesium cernuum* L.

**DOI:** 10.1155/2021/5515961

**Published:** 2021-04-29

**Authors:** Yuan-she Huang, Jing-xin Mao, Lai Zhang, Hong-wei Guo, Chen Yan, Min Chen

**Affiliations:** ^1^College of Pharmaceutical Sciences, Southwest University, Chongqing 400715, China; ^2^Anshun College, Anshun Guizhou 561000, China; ^3^An Shun City People's Hospital, Anshun 561000, China

## Abstract

**Objective:**

The aim of the study was to investigate the antiprostate cancer effects and mechanism of ineupatolide (T-21), a natural product isolated from the Compositae plant *Carpesium cernuum* L., on PC-3 human prostate cancer cells.

**Methods:**

The effect of T-21 on the proliferation of PC-3 cells was detected by 3-(4,5-dimethylthiazol-2-yl)-2,5-diphenyltetrazolium bromide, cell migration, and invasion experiments; the morphology of cell apoptosis was observed by Hoechst-propidium iodide staining; the effects of T-21 on PC-3 cell apoptosis and the cell cycle were evaluated by flow cytometry; and the effect of T-21 on the expression levels of phosphorylated protein kinase B (p-AKT), AKT, X-linked inhibitor of apoptosis protein (xlAP), procaspase-3, and poly (ADP-ribose) polymerase (PARP) in PC-3 cells was measured by western blotting.

**Results:**

T-21 significantly inhibited the proliferation of cells, and its half-maximal inhibitory concentrations at 12, 24, and 48 h were 38.46 ± 1.01, 24.63 ± 0.70, and 7.36 ± 0.58 *μ*M, respectively. T-21 may promote cell apoptosis in a concentration-dependent manner and block the cell cycle in the G2 and S phases. In addition, T-21 significantly reduced the protein expression levels of p-AKT, AKT, xlAP, procaspase-3, and PARP.

**Conclusion:**

T-21 exhibits antiproliferation effects on PC-3 cells by promoting apoptosis and arresting the cell cycle in the G2 and S phases. The possible mechanism underlying its potential therapeutic effects against prostate cancer is related to the AKT/xlAP pathway.

## 1. Introduction

Prostate cancer, which ranks second in the global incidence of male cancers and sixth in mortality, is currently one of the diseases with the highest mortality in middle-aged and elderly men around the world [1]. In European and American countries, the number of deaths caused by prostate cancer accounts for a significant number of deaths caused by malignant tumors, second only to lung cancer [2]. The incidence of prostate cancer gradually increases with age. However, researchers have yet to determine the exact cause of prostate cancer, which may be related to the environment, heredity, and sex hormones [3]. With the development of the disease, the urethra is gradually compressed by the prostate, which may cause dysuria, sexual dysfunction, and hematuria [4]. The onset of prostate cancer is relatively insidious, and early diagnosis is very difficult; thus, the tumor has often metastasized by the time it is discovered [5]. In terms of clinical diagnosis, most patients are already at an advanced stage, with local invasion and distant metastasis. In these cases, the effect of surgery is not ideal, or the opportunity for radical surgery has already been lost [6, 7].

The article "Antiprostate Cancer Activity of Ineupatolide Isolated from Carpesium cernuum L" was published in 2021. Journal: Biomed Res Int.

Natural products are known to exert certain anticancer effects, such as promoting tumor cell apoptosis, inhibiting tumor cell proliferation, and inducing tumor cell differentiation. Owing to their unique advantages, natural medicines play an important role in the treatment of human cancer and have great developmental potential. According to statistics, between 1939 and 2016, 50% of the new drugs approved by the U.S. Food and Drug Administration were directly or indirectly derived from natural products [8]. Therefore, it is of great significance to develop new drugs from natural products.

*Carpesium* L. is a perennial herb of the Compositae family. There are 18 species and 3 varieties *of Carpesium* L. in China, which are mainly distributed in the southwest areas [9]. Among them, *Carpesium abrotanoides* Linn., *Carpesiu*m *divaricatum* Sieb. et Zucc., *Carpesium macrocephalum* Franch. et Sav., *Carpesium lipskyi* Winkl., *Carpesium nepalense* Less. var. nepalense, *Carpesium nepalense* Less var. lanatum, *Carpesium cernuum* L., *Carpesium minum* Hemsl., *Carpesium triste* Maxim., *Carpesium faberi* Winkl., *Carpesium longifolium* F. H. Chen et C. M. Hu, and *Carpesium trachelifolium* Less. were reported be used for medicinal purposes, including detoxifying, expectorating, and stopping bleeding [10].

Previous studies have shown that *Carpesium cernuum* L. contains a variety of chemical components, some of which exhibit different antitumor, anti-inflammatory, antioxidant, and immunomodulatory effects [11–13]. In addition, it has been reported that the primary chemical components of *Carpesium cernuum* L. are terpenoids and flavonoids [14]. Whether this plant can be utilized as a new human antitumor substance urgently requires further research. The results of a previous study showed that the compound ineupatolide (T-21) exhibits the activities of antitumor in the cell experiment [15]. However, information on the pharmacological activity and antitumor mechanism of T-21 in PC-3 cells has not yet been reported. Therefore, this study was aimed at investigating the antiprostate cancer effects and underlying mechanism of the action of T-21.

The article "Antiprostate Cancer Activity of Ineupatolide Isolated from Carpesium cernuum L" was published in 2021. Journal: Biomed Res Int.

## 2. Material and Methods

### 2.1. Chemicals and Reagents

The entire plant of *Carpesium cernuum* L. was collected from Zhenning, Guizhou Province, and identified by professor Min Chen at Southwest University College of Pharmaceutical Sciences. T-21 was extracted from the ethyl acetate part of *Carpesium cernuum* L. and refined into medicinal material with purity > 98% (Figure 1(a)). The primary extraction, isolation, and purification of T-21 were shown as follows: powder of the air-dried roots (5 kg) of *Carpesium cernuum* L. was extracted by maceration with 95% ethanol overnight at room temperature. The ethanol extract was evaporated in vacuo to yield a semisolid (0.54 kg), which was suspended in water (5 L) and partitioned with petroleum ether (15 L), ethyl acetate (15 L), and n-butanol (15 L), successively. The ethyl acetate solution was concentrated to yield 316 g of residue, which was subjected to silica gel chromatography (100∼200 meshes, 70 cm × 10 cm, ID) and eluted with petroleum ether ethyl acetate mixtures of increasing polarity (99 : 1 to 10 : 1) to obtain a total of 16 fractions. T-21 was obtained from fraction 6 (Fr. 6), and Fr. 6 (21.3 g) was separated continuously to obtain T-21 (12.6 mg). Finally, based on the physical and spectral data, it was identified as T-21. A 3-(4,5-dimethylthiazol-2-yl)-2,5-diphenyltetrazolium bromide (MTT) kit, mycin-streptomycin solution, dimethyl sulfoxide (DMSO) solution, Tween 20, an 8 *μ*m pore size transwell chamber, a flow cytometry kit, a fluorescein isothiocyanate apoptosis kit, and an annexin kit were purchased from Beyotime Biotechnology Co., Ltd. (Shanghai, China). Crystal violet staining solution, trypsin, low-sugar Dulbecco's Modified Eagle's Medium (DMEM), and fetal bovine serum (FBS) were purchased from Invitrogen (Carlsbad, CA, USA). Mouse anti-human phosphorylated protein kinase B (p-AKT), AKT, X-linked inhibitor of apoptosis protein (xlAP), procaspase-3, poly (ADP-ribose) polymerase (PARP), glyceraldehyde 3-phosphate dehydrogenase (GAPDH), and horseradish peroxidase-labeled goat anti-rabbit immunoglobulin G antibodies as well as an electrochemiluminescence (ECL) kit were purchased from Cell Signaling Technology (Danvers, MA, USA). Glutaraldehyde, osmic acid, anhydrous acetone, epoxy resin, uranyl acetate, and lead citrate were purchased from Beijing Zhongjing Technology Co., Ltd. (Beijing, China).

### 2.2. Cell Culture

PC-3 cells were purchased from the Shanghai Institute of Cell Biology, Chinese Academy of Sciences (Shanghai, China). The PC-3 cells were placed in DMEM containing 10% FBS, 100 *μ*g/mL streptomycin, and 100 U/mL penicillin and then cultured in an incubator at 37°C with 5% CO_2_. When the cells grew to the monolayer cell flask, they were digested by pipetting with 0.25% trypsin into a single-cell suspension and passaged at a ratio of 1 : 3. The cells were passaged once every 2 to 3 days.

The article "Antiprostate Cancer Activity of Ineupatolide Isolated from Carpesium cernuum L" was published in 2021. Journal: Biomed Res Int.

### 2.3. Hoechst 33258 Staining

PC-3 cells were seeded into a 6-well culture plate, and the experiment was divided into 4 groups: (1) control group: normal control; (2) low concentration group: with concentration of 10 *μ*M T-21; (3) medium concentration group: with concentration of 20 *μ*M T-21; and (4) high concentration T-21 group: with concentration of 40 *μ*M T-21. After each group was cultured for 24 h, the cells were collected. Each well was fixed with 4% paraformaldehyde for 20 min, washed with phosphate-buffered saline (PBS), stained with Hoechst 33258 fluorescent dye solution at room temperature for 15 min, washed again with PBS, and placed under a fluorescent microscope to observe the morphological changes of PC-3 cells and take pictures.

### 2.4. Cell Viability Assay

PC-3 cells were inoculated into a 96-well plate with 200 *μ*L/well after adjusting the cell density to 5 × 10^4^ mL^−1^. After cell culture in a 37°C and 5% CO_2_ incubator for 24 h, the culture medium was replaced with 200 *μ*L of DMEM and 5, 10, 20, 40, or 80 *μ*M of T-21 in each well. A negative control group (containing equal volumes of DMEM and DMSO) with six replicate wells for each concentration was set up. After incubation for 24, 48, or 72 h, 20 *μ*L of an MTT/phenazine methosulfate mixture was added to each well, and the cells were incubated for another 3 h. A microplate reader was used to measure the absorbance value of each well at a wavelength of 450 nm, and the cell proliferation inhibition rate and half-maximal inhibitory concentration (IC_50_) were calculated using GraphPad Prism 6.0 software (GraphPad Software, San Diego, CA, USA).

### 2.5. Cell Morphology

After digestion, the cells in each group were transferred to a 10 mL centrifuge tube, centrifuged, fixed before adding 2.5% glutaraldehyde, fixed again after adding 1% osmic acid, dehydrated, embedded in anhydrous acetone plus epoxy resin for 2 h, cut into 70–80 nm ultrathin sections, stained with uranyl acetate and lead citrate, observed, and photographed under a transmission electron microscope.

### 2.6. Apoptosis and Cell Cycle Assays

PC-3 cells were collected and seeded into a 6-well culture plate at a density of 8 × 10^5^ cells/well. After cell culture for 12 h using 10, 20, or 40 *μ*M T-21 to treat the cells, an equal volume of DMSO was added to the control group. After culturing for another 24 h, the cells were collected. For the detection of cell apoptosis, 2 *μ*L of propidium iodide (PI) staining solution, 2 *μ*L of annexin V staining solution, and 300 *μ*L of PBS were added to each group of samples, followed by flow cytometry analysis. For detection of the cell cycle, 300 *μ*L of Reagent A solution and 2 *μ*L of Reagent B solution were added to each group of samples, mixed, and incubated in the dark for 30 min, and then, flow cytometry analysis was performed. We used Cell ModFit software for statistical analysis of the data.

The article "Antiprostate Cancer Activity of Ineupatolide Isolated from Carpesium cernuum L" was published in 2021. Journal: Biomed Res Int.

### 2.7. Western Blotting

PC-3 cells were treated with 10, 20, or 40 *μ*M T-21 for 24 h, resuspended, and centrifuged at 7000 rpm for 10 min. The cells were then collected and washed twice with precooled PBS. After lysis with the precooled cell lysate, the supernatant was collected, and the protein concentration of each sample was determined. Following protein quantification, 50 *μ*g of protein was added to the loading buffer and denatured at 95°C for 10 min. After sodium dodecyl sulfate polyacrylamide gel electrophoresis, transfer, and blocking, 1 : 200 dilutions of p-AKT, AKT, xlAP, procaspase-3, and PARP primary antibodies were added and incubated overnight at 4°C. Next, the secondary antibody (1 : 1000) was added and incubated for 1 h at room temperature. The membrane was washed three times with Tris-buffered saline-Tween 20, fixed, and photographed using ECL. ImageJ software (National Institutes of health, Bethesda, MD, USA) was used for grayscale analysis.

### 2.8. Scratch Cell Migration Assay

PC-3 cells were cultured overnight upon seeding on a 6-well plate at a density of 3 × 10^5^ cells/well. After comparing the center line of the 6-hole plate with a ruler, horizontal lines were drawn vertically on the cell surface with 10 *μ*L of sterile gun head. Three horizontal lines and one vertical line were drawn for each hole. The cells were washed three times with PBS to remove the serum and marked cells. Next, the drug-containing serum-free medium was added, recorded as 0 h, and photographed. After taking the picture, the 6-well plate was kept in a CO_2_ incubator for cultivation, and another picture was taken 48 h later. The positions of the blank area at 0 and 48 h and the migration rate were calculated.

### 2.9. Transwell Cell Invasion Assay

Matrigel was diluted with serum-free medium at a ratio of 1 : 40 to a concentration of 200–300 *μ*g/mL. A precooled sterile pipette tip was used to absorb the diluted Matrigel and spread it in a 100 *μ*L transwell chamber, which was then placed in a 37°C incubator for approximately 2 h to make the Matrigel form a thin film. The serum-free medium was subsequently removed from the chamber, the PC-3 cells were resuspended, the cell density was adjusted to 10^5^ cells/mL, and 200 *μ*L of cell suspension was added to each well of the upper chamber. Next, 500 *μ*L of medium containing 10% FBS was added to the lower chamber, which was placed in a CO_2_ incubator for 16–20 h. Thereafter, the medium in the upper chamber was dried, the cells in the upper layer of the chamber were removed with a cotton swab, and the chamber was placed in 4% paraformaldehyde for 20 min of fixation. The chamber was stained with 1% crystal violet staining solution for 30 min, washed with PBS buffer 3 times after removing any excess crystal violet, and placed under an inverted microscope to be photographed.

The article "Antiprostate Cancer Activity of Ineupatolide Isolated from Carpesium cernuum L" was published in 2021. Journal: Biomed Res Int.

### 2.10. Data Analysis

The data are presented as means ± standard deviations. The comparison between groups was performed using a one-way analysis of variance and the least significant difference test for statistical analysis of each data point (GraphPad Prism 5.0 software; GraphPad Software). *P* < 0.05 or *P* < 0.01 were considered to indicate statistical significance.

## 3. Results

### 3.1. Effect of T-21 on the Proliferation of PC-3 Cells

The cell proliferation assay results are shown in Figure 1. Compared to the control group, as the exposure time and T-21 concentration increased, the cell proliferation inhibition rate in the treated groups gradually increased (Figure 1(b)). The growth of PC-3 cells in each concentration group was significantly inhibited with the increases in exposure time and T-21 concentration (Figure 1(c)). The IC_50_ values were 38.46 ± 1.01, 24.63 ± 0.70, and 7.36 ± 0.58 *μ*M at 24, 48, and 72 h, respectively (Figure 1(d)).

### 3.2. Effect of T-21 on PC-3 Cell Apoptosis

The results of Hoechst-PI staining are shown in Figure 2(a). The nuclei of the control group were uniformly stained with low fluorescence intensity. Concentrated chromosomes and apoptotic bodies appeared in the cells at each concentration of T-21, the cell density decreased, and the fluorescence intensity increased significantly, indicating that T-21 can induce PC-3 cell apoptosis. The results of flow cytometry are shown in Figures 2(b) and 2(c). Compared to the control group, treatment with 10, 20, or 40 *μ*M T-21 for 24 h significantly induced PC-3 cell apoptosis, and the apoptosis rate was significantly different (*P* < 0.05 and *P* < 0.01). The apoptotic rate in the high concentration group was 18.33 ± 1.75, and there was a clear dependence on concentration.

### 3.3. Effect of T-21 on the Cell Cycle

The cell cycle analysis results are shown in Figures 2(d) and 2(e). After treating PC-3 cells with 10, 20, or 40 *μ*M T-21 for 24 h, compared to the control group, the proportions of cells in the G1 phase, G2 phase (13.08 ± 0.28, 13.66 ± 1.12, 14.22 ± 0.26, and 21.00 ± 1.06, respectively), and S phase (10.24 ± 0.39, 10.37 ± 0.31, 9.68 ± 0.11, and 19.35 ± 0.23, respectively) of each group increased with the dose concentration. There were obvious gradient changes (*P* < 0.05 and *P* < 0.01), the cells in the G1 phase gradually decreased, and the cells in the G2 and S phases gradually increased, indicating that T-21 can significantly block the cell cycle in the G2 and S phases.

The article "Antiprostate Cancer Activity of Ineupatolide Isolated from Carpesium cernuum L" was published in 2021. Journal: Biomed Res Int.

### 3.4. Effect of T-21 on the Expression Levels of Related Proteins in the AKT/xlAP Signaling Pathway in PC-3 Cells

The results are shown in Figure 3. After treating PC-3 cells with 10, 20, or 40 *μ*M T-21 for 24 h, the expression levels of p-AKT, AKT, xlAP, procaspase-3, and PARP gradually decreased. These results demonstrate a significant effect of promoting PC-3 cell apoptosis, which may be related to the downregulation of the expression levels of AKT/xlAP pathway-related proteins.

### 3.5. Effect of T-21 on the Migration Ability of PC-3 Cells

To explore the effect of T-21 on the migration ability of PC-3 cells, the scratch area of cells before and after treatment with 10, 20, or 40 *μ*M T-21 for 48 h was analyzed. As shown in Figures 4(a) and 4(b), compared to 0 h of drug treatment, after 24 h and 48 h, the scratch areas of the T-21 0, 10, 20, and 40 *μ*M treatment groups were 55%, 80%, 94%, and 60.8% and 1%, 36%, 62%, and 79%, respectively. These results indicate that T-21 exerts a dose-dependent and time-dependent inhibitory effect on PC-3 cell migration.

### 3.6. Effect of T-21 on the Invasion Ability of PC-3 Cells

The invasion assay results are shown in Figures 4(c) and 4(d). After treating PC-3 cells with 10, 20, or 40 *μ*M T-21 for 16 h, compared to the control group, the proportion of cells passing through Matrigel was 76.8%, 73.6%, and 51.1%, respectively. These results suggest that T-21 administration may have a significant impact on the invasion ability of PC-3 cells.

## 4. Discussion

Prostate cancer is one of the male malignant tumors that has rapidly increased in incidence in China in recent years [16]. It has been reported that prostate cancer patients are prone to bone metastasis and severe bone pain in the advanced stage, which seriously affects their quality of life [17]. Previous studies have shown that the current treatment effect for prostate cancer patients is not ideal, and its high fatality and recurrence rates are closely related to the high metastasis and invasion ability of prostate cancer cells [18]. In recent years, research on the mechanism of antitumor metastasis has progressed, and an increasing number of action sites that can be used to block tumor metastasis have been identified, which provides a broad avenue for the development of antitumor metastasis drugs [19].

The article "Antiprostate Cancer Activity of Ineupatolide Isolated from Carpesium cernuum L" was published in 2021. Journal: Biomed Res Int.

Traditional Chinese medicine has great advantages and is used as an adjuvant treatment for prostate cancer surgery, radiotherapy, and chemotherapy [20]. It has been discovered that natural products may exert antitumor effects in a variety of ways, such as inhibiting tumor cell proliferation, infiltration, and metastasis as well as inducing differentiation, cell apoptosis, and antitumor cell adhesion [21]. In the present study, it was found that T-21 may inhibit the growth of PC-3 cells in a dose-dependent manner after treating the cells with 10, 20, or 40 *μ*M T-21 for 24 h. Hoechst fluorescence staining demonstrated that T-21 can induce PC-3 cells to undergo typical nuclear fragmentation, showing dense granular fluorescence. The effects of T-21 on PC-3 cell proliferation and apoptosis were also studied, which showed that with an increase in T-21 concentration, the inhibition rate of PC-3 cell proliferation increased, the proportion of early and late apoptotic cells increased significantly, and the G2 and S phases of the cell cycle were clearly blocked, collectively indicating that T-21 exerts antitumor activity against PC-3 cells *in vitro*.

The results of the present study showed that T-21 significantly promotes the apoptosis of PC-3 cells, which may be related to the downregulation of the expression levels of AKT/xlAP pathway-related proteins. Previous studies have shown that AKT is a downstream target protein of phosphoinositide 3-kinase in the signal transduction pathway, and its continuous activation is closely related to the occurrence and development of tumors [22]. It has also been reported that AKT expression is often overexpressed in many cancers, such as pancreatic cancer, breast cancer, and non-small-cell lung cancer [23–25]. Previous research has suggested that when AKT is mutated, the mobility of cells is also reduced, indicating that AKT plays an important role in tumor migration and invasion [26]. In addition, the activation of p-AKT has been found to play an important role in the transition from the G1 phase to the S phase of the cell cycle, thereby promoting cell proliferation [27].

It has previously been demonstrated that there is a high concentration of phosphorylated AKT protein in the tumor cells of prostate cancer patients and that procaspase-3 is involved in the entire process of cell apoptosis [28]. Furthermore, inactive procaspase-3 and active cleaved caspase-3 exist in the cytoplasm. When procaspase-3 is cleaved, two subunits, p17 and p12, remain active [29]. After cleaved caspase-3 begins its protease journey, it can cleave the downstream PARP and other substrates, thereby exerting its role in promoting apoptosis [30]. PARP is a DNA repair enzyme and the cleavage substrate of caspase, the core member of apoptosis, which plays an important role in DNA damage repair and cell apoptosis [31]. Previous studies have shown that inhibiting the expression of PARP in cells has a significant inhibitory effect on cell proliferation and induces cell apoptosis [32]. Recent studies have also suggested that xlAP participates in regulating cell apoptosis by inhibiting caspase activity in prostate cancer and other malignant tumors [33].

The article "Antiprostate Cancer Activity of Ineupatolide Isolated from Carpesium cernuum L" was published in 2021. Journal: Biomed Res Int.

Taken together, the present study indicates that T-21 exhibits antiproliferation effects in PC-3 cells by promoting apoptosis and arresting the cell cycle in the G2 and S phases. The possible underlying mechanism of its potential therapeutic effects against prostate cancer is related to the AKT/xlAP pathway.

## Figures and Tables

**Figure 1:** Effects of T-21 on PC-3 cell morphology and survival. (a) Structure of T-21 isolated from *Carpesium cernuum* L. (b) Morphology of PC-3 cells after treatment with T-21 for 24 h. (c) PC-3 cells induced by T-21 (0, 10, 20, or 40 *μ*M) were treated for 24 h and detected using the 5-ethynyl-2′-deoxyuridine method. The cell images were captured at a magnification of 100× (scale: 100 *μ*m). (d) Cytotoxicity of T-21 against PC-3 cells (MTT assay; IC_50_ values). PC-3 cells were treated with T-21 (5–80 *μ*M) at different concentrations for 24, 48, or 72 h. The data are presented as means ± standard deviations (*n* = 3). ^∗^*P* < 0.05 and ^∗∗^*P* < 0.01 vs. the control group.

**Figure 2:** Effects of T-21 on the apoptosis and cell cycle of PC-3 cells. (a) PC-3 cells were treated with T-21 for 24 h, fixed, and stained with Hoechst. Nucleus changes and the formation of apoptotic bodies were observed using a fluorescence microscope (10 × 40). (b, c) T-21 (10, 20, or 40 *μ*M) was used to treat PC-3 cells for 24 h, which were then were fixed and stained with annexin V/PI. Flow cytometry was used to detect and analyze cell apoptosis in each group. The data are presented as means ± standard deviations (SDs; *n* = 3). ^∗^*P* < 0.05 and ^∗∗^*P* < 0.01 vs. the control group. (d, e) PC-3 cells were treated with T-21 (10, 20, or 40 *μ*M) for 24 h, fixed, and stained with PI. DNA content was detected and analyzed by flow cytometry. The percentage of PC-3 cells at different stages of the cell cycle is demonstrated by the bar graph. The data are presented as means ± SDs (*n* = 3). ^∗^*P* < 0.05 and ^∗∗^*P* < 0.01 vs. the control group.

**Figure 3:** Effects of T-21 on the AKT/xlAP signaling pathway of PC-3 cells. T-21 (10, 20, or 40 *μ*M) was used to treat PC-3 cells for 24 h, after which total protein was extracted. (a) The expression levels of apoptotic pathway-related proteins were detected by western blotting in PC-3 cells treated with T-21. (b–e) Quantitative analysis of protein expression levels using ImageJ software (National Institutes of Health). GAPDH was used as an internal reference control protein. Data are presented as means ± SDs (*n* = 3). ^∗^*P* < 0.05 and ^∗∗^*P* < 0.01 vs. the control group.

The article "Antiprostate Cancer Activity of Ineupatolide Isolated from Carpesium cernuum L" was published in 2021. Journal: Biomed Res Int.

**Figure 4:** Effects of T-21 on the migration and invasion abilities of PC-3 cells. (a, b) The scratch areas of PC-3 cells before and after treatment with 10, 20, or 40 *μ*M T-21 for 48 h were analyzed to determine the cell migration ability. (c, d) PC-3 cell treatment with 10, 20, or 40 *μ*M of T-21 for 16 h. The data are presented as means ± standard deviations (*n* = 3). ^∗^*P* < 0.05 and ^∗∗^*P* < 0.01 vs. the control group.

## Data Availability

The data used to support the findings of this study are available from the corresponding author upon request.
